# Effect of Acupuncture on Polycystic Ovary Syndrome in Animal Models: A Systematic Review

**DOI:** 10.1155/2021/5595478

**Published:** 2021-09-24

**Authors:** Yan Li, Lijia Zhang, Jinjin Gao, Jun Yan, Xue Feng, Xiting He, Hong Jin, Xinyu Li, Zhengyi Cui, Junfei Zhao, Fengyi Liu, Xiaowai Liu, Yongfei Liu, Wan Ren, Songjiang Liu

**Affiliations:** ^1^First Affiliated Hospital, Heilongjiang University of Chinese Medicine, 26 Heping Road, Harbin 150040, China; ^2^Heilongjiang University of Chinese Medicine, 24 Heping Road, Harbin 150040, China

## Abstract

**Background:**

Polycystic ovary syndrome (PCOS) is one of the most common endocrine disorders among women of reproductive age. As a widely used complementary and alternative therapy, acupuncture is increasingly used to treat PCOS. However, the effect of acupuncture in treating PCOS is uncertain, and the mechanisms are unclear. This systematic review aims to determine the efficacy of acupuncture on PCOS in animal preclinical models.

**Methods:**

Experimental animal studies of acupuncture in PCOS animal models were searched in PubMed, Web of Science, China National Knowledge Infrastructure, and the Chinese Science and Technology Periodical Database from inception to December 2020. The risk of bias was assessed using the Systematic Review Centre for Laboratory Animal Experimentation (SYRCLE) risk of bias tool.

**Results:**

A total of 358 studies were screened based on the title and abstract, and 31 studies were included. A total of 722 animals were involved, and all studies used either Wistar rats or SD rats. Twenty-six studies used electroacupuncture, 9 studies used manual acupuncture, and 5 of them employed both electroacupuncture and manual acupuncture. A total of 22 acupoints were involved; 7 studies followed the modern acupuncture pattern, and the rest followed classic acupuncture theory.

**Conclusions:**

The present review summarizes the current evidence of the effects of acupuncture on PCOS in animal models. Unfortunately, we could not draw a definite conclusion due to the methodological weakness of the included studies and the high heterogeneity. Well-designed studies are needed in the future to fill this gap.

## 1. Introduction

Polycystic ovary syndrome (PCOS) is a heterogeneous endocrine disorder among females of reproductive age. The worldwide prevalence of PCOS is 8–13% in women and 6% in adolescent girls [1–3]. Its clinical manifestations are diverse and characterized by irregular menstruation, amenorrhea, androgen excess, chronic anovulation, and infertility. Fifty percent of women with PCOS have insulin resistance (IR) [4], which is associated with an increased risk of metabolic syndrome, type 2 diabetes, and cardiovascular diseases [5]. The pathogenesis of PCOS is not fully understood. In recent years, an increasing number of studies have found that disorders of the hypothalamus-pituitary-ovarian (HPO) axis, abnormal adrenocortical function, and enhanced sympathetic nerve activity are all involved in PCOS development [6–8].

As the prevalence of PCOS increases, studies of effective treatment regimens are particularly important. Acupuncture is an important part of traditional Chinese medicine that has been applied for thousands of years. Some clinical studies found that acupuncture is beneficial for the regulation of hormone levels and ovulatory dysfunction in patients with PCOS [9–11]. Several systematic reviews have been conducted on the efficacy and safety of acupuncture for women with PCOS, but due to the high risk of bias and heterogeneity, the levels of evidence are low [12]. There is an insufficient amount of research evidence to support the clinical efficacy of acupuncture treatment for women with PCOS. Preclinical animal experiments are the link between basic research and clinical trials. Several animal experimental studies indicate that acupuncture influences PCOS-like symptoms in rats via multiple mechanisms [13, 14]. Peng et al. [13] found that acupuncture can improve insulin resistance by activating the AMPK pathway in PCOS-like symptoms. Xu et al. [14] indicated that acupuncture adjusts hormone levels by regulating ovarian local factors in PCOS rats.

Until now, no systematic review has been published to summarize the effects of acupuncture in PCOS animal models. This systematic review of animal experiments is an efficient means of enhancing the value of animal experiments, which reduces the risk of the translation of animal experiments to the clinic. Therefore, this systematic review aimed to evaluate the currently available evidence of acupuncture in PCOS animal models and provide valuable directions to inform clinical practice.

## 2. Materials and Methods

### 2.1. Protocol and Registration

The protocol of this study followed the preferred reporting items for systematic reviews and meta-analysis (PRISMA) guidelines (Additional file 1) [15] and is adapted from the structure provided in the Systematic Review Protocol for Animal Intervention Studies [16]. This study was registered at OSF (Registration DOI: 10.17605/OSF.IO/FNM37).

### 2.2. Eligibility Criteria

#### 2.2.1. Types of Studies Included

This systematic review included both randomised and nonrandomised controlled studies. There was no restriction on language or date. We included studies published in peer-reviewed journals only [17].

#### 2.2.2. Types of Animal Models

All animal models of PCOS were included regardless of the species or size of the animal.

#### 2.2.3. Types of Intervention and Comparators

Both traditional acupuncture and contemporary acupuncture (in which needles were not inserted in classical meridian points) were included. Hand stimulation, electrical stimulation, or warming needles with moxibustion were included. Acupuncture without needling was excluded, such as acupressure, acupoint injection, tap pricking, and cupping. The comparison group included PCOS animals induced by the same method as the intervention group but without undergoing the intervention [17].

#### 2.2.4. Types of Outcome Measures

The following outcome measures were used [17]:

1. Primary outcome: homeostatic model assessment-insulin resistance (HOMA-IR: (fasting insulin (*μ*U/mL) × fasting glucose (mmol/L))/22.5).
2. Secondary outcomes: testosterone (T), LH (luteinizing hormone), LH/follicle-stimulating hormone (FSH) ratio, fasting blood sample (FBG), fasting insulin (FINS), and body weight (BW).

### 2.3. Search Strategy

PubMed, Web of Science, China National Knowledge Infrastructure (CNKI), and the Chinese Science and Technology Periodical Database (VIP) were searched from inception to December 20, 2020. The main terms “Polycystic ovary syndrome”, “Acupuncture”, and “Animal Experimentation”, indexed in the MeSH system, were combined [17].

### 2.4. Study Selection

Two independent reviewers (JY and LJZ) screened titles and abstracts for eligibility. Disagreements between reviewers were resolved by a third review (YL). Full texts were obtained and evaluated by the same reviewers using a predesigned form.

### 2.5. Data Extraction

Two reviewers (JY and LJZ) extracted data independently, and any controversy was resolved by discussion. The following information was recorded using a predesigned form: study design, characteristics of the included animals, characteristics of the animal model, details of the intervention, and outcome measures.

### 2.6. Risk of Bias Assessment

Two reviewers (YL and JJG) assessed the risk of bias using SYRCLE's tool for assessing risk of bias (SYRCLE ROB) [18].

### 2.7. Data Synthesis

We performed a meta-analysis using a random-effects model with Review Manager (RevMan) 5.3. Treatment effects were summarized as the standard mean difference (SMD) with a 95% confidence interval (CI). The SMD is an evaluation of the combined effect sizes, and *P* values below 0.05 were considered statistically significant. The presence of heterogeneity was evaluated by *I*^2^ and chi-square statistical analyses. Funnel plots were performed to evaluate publication bias if there were more than ten studies included [17].

## 3. Result

### 3.1. Study Selection

A total of 384 potentially relevant studies were identified from the abovementioned four databases. After removing duplicates, 358 records remained for title and abstract screening. A total of 303 studies were excluded due to at least one of the following reasons: (1) not an animal study, (2) case report or review, or (3) not related to acupuncture. Finally, 55 studies remained after the initial reading. After full-text reading of the remaining studies, 24 studies were excluded, and 31 studies were included (Figure 1).

### 3.2. Study Characteristics

A total of 31 studies were included [13, 14, 19–46]. Thirteen studies were published in English, and 18 were published in Chinese. A total of 722 animals (9 studies with Wistar rats and 22 studies with SD rats) were involved, and the details of the animal models are presented in Table 1. Eleven studies induced a PCOS model by letrozole, 8 studies used dihydrotestosterone (DHT), 6 studies used dehydroepiandrosterone (DHEA), 4 studies used testosterone propionate (TP), 1 study used estradiol valerate (EV), and 1 study used prasterone sulfate. Thirty included studies randomly assigned animals to the acupuncture and control groups, and only 1 study did not report randomisation details. Twenty-six studies used electroacupuncture (EA), 9 studies used manual acupuncture (MA), and 5 of them employed two acupuncture groups, including both EA and MA. Among all the included studies, a total of 22 acupoints were involved. The frequencies of acupuncture points from high to low were as follows: SP6, 20 times; CV4 (RN4), 17 times; CV3 (RN3), 10 times; ST36, 7 times; EX-CA1, 7 times; ST29, 4 times; RN12, 3 times; ST25, 3 times; LI10, 2 times; BL23, 2 times; SP9, 1 time; ST40, 1 time; RN6, 1 time; PC6, 1 time; EX-B3, 1 time; CV12, 1 time; BL18, 1 time; BL20, 1 time; ST27, 1 time; ST28, 1 time; LR3, 1 time; and Hou Hui, 1 time. Seven studies followed the modern acupuncture pattern, in which the basic principle was two needles inserted bilaterally in the abdominal muscles, with two needles placed in each soleus and gastrocnemius hindlimb muscle in somatic segments corresponding to ovarian innervations [18, 19, 23, 24, 26, 31, 36]. The electrical frequencies used were all 2 Hz except for one study that did not mention the EA frequency, and the intensity was 0.6–3 mA. One study reported intervention with a single session; the others lasted from 2 weeks to 8 weeks.

### 3.3. Risk of Bias within Studies

The results of the risk of bias of the included studies are summarized in Table 2. SYRCLE ROB included domains for selection bias (sequence generation, baseline characteristics, and allocation concealment), performance bias (random housing and blinding), detection bias (random outcome assessment and blinding), attrition bias, reporting bias, and other biases.

### 3.4. Effectiveness

The meta-analysis was not performed since the heterogeneity was significantly high. Although the heterogeneity analysis was carried out based on sensitivity analysis, the detailed reasons for the potential heterogeneity were not very certain.

### 3.5. Quality of Evidence Assessment (Table 3)

The GRADE recommendations for HOMA-IR, T, FINS, and BW were very low, and those for LH, LH/FSH, and FBG were low. The certainty was downgraded for the following reasons: I values that exceeded 75%; different animal modelling methods; differences in the treatment cycle and dosage; physiological and pathological differences between rodents and humans; small sample size; and the 95% CI included the value of one.

## 4. Discussion

### 4.1. Summary of Evidence

To the best of our knowledge, this is the first systematic review summarizing the current evidence of the effects of acupuncture on PCOS in animal experiments. This finding suggests that acupuncture may play a potential role in restoring reproductive endocrine function in PCOS-like animal models.

The mechanisms of acupuncture in PCOS animal models are still unclear. It is well known that elevated sympathetic activity contributes to the development and maintenance of PCOS [47, 48]; thus, the sympathetic nervous system may offer a novel therapeutic target in treating PCOS. Normal ovulation requires three components, namely, an intact central hypothalamic-pituitary-ovarian axis, synchronized feedback signals, and normal local responses within the ovary [49]. The evidence suggests that low-frequency EA could lower sympathetic activity, and the effects may be mediated by modulation of NGF expression of sympathetic outflow to the ovaries in PCOS-like rats [50]. Zhang et al. reported that the regulation of EA in reproductive function in PCOS-like rats may not be accomplished by the hypothalamic-pituitary-ovarian axis [22, 23], while Maliqueo et al. reported that low-frequency EA significantly affects the pituitary-ovarian axis by normalizing LH secretion [32]. This contradiction is likely due to different PCOS-like rat models and the different forms of acupuncture employed and it needs to be elucidated with further experiments. It has now been demonstrated that the effect of low-frequency EA on ovarian function is mediated as a reflex response via the ovarian sympathetic nerves, and the response is controlled via supraspinal pathways [51]. It has been newly demonstrated that ovarian innervation likely plays an important role in folliculogenesis, and EA might restore PCOS pathophysiology by regulating ovarian innervation, at least partially mediated through the superior ovarian nerve. The effect of EA is based on the integrity of the nervous system [46].

Other hypotheses have also been reported. EA stimulates the development and maturation of eggs in PCOS-like rats by increasing the level of stem cell factor and reducing the level of TNF-*α* responsible for follicular fluid [26]. EA could increase P450arom and decrease P450c17*α* as well as the expression levels of their mRNA in ovarian tissues in PCOS-like rats. These effects may thereby change the local ovarian environment of excessive androgen and improve the reproductive, endocrine, and metabolic disorders associated with PCOS [28]. Adiponectin reduces androstenedione synthesis in human theca cells [52]. EA stimulated the ovarian adiponectin system in rats with letrozole-induced PCOS, and the effect does not seem to be mediated by modulation of sympathetic activity [32]. Oxidative stress is now recognized to play a central role in the pathophysiology of PCOS [53]. Zheng et al. reported that EA decreases serum malondialdehyde levels and increases superoxide dismutase levels, hence improving the oxidative stress status of PCOS-like rats [33]. EA not only regulates abnormal glucose and lipid metabolism in PCOS-like rats but also increases glucose transporter 1 and glucose transporter 4 expression in ovarian tissue, which may alleviate insulin resistance [35]. EA increases angiogenesis in the antral follicles of PCOS-like rats, which favours follicle maturation, and ovulation is suggested as being one of the mechanisms involved in the effects of EA on PCOS [54]. It has also been demonstrated that EA regulates androgen receptor and Connexin 43 (which plays an important role in the process of oocyte meiosis and follicular selection) in PCOS-like rats; however, further studies are needed to clarify whether this is one of the mechanisms involved in the effects of EA on PCOS [14]. It has recently been recognized that autophagy is involved in the occurrence and development of PCOS [55]. Huang et al. demonstrated that EA inhibits autophagy in ovarian tissue through the PI3K/AKT pathway [44]. Sterol regulatory element binding protein-1 (SREBP1) is a key gene in lipid metabolism regulation. Peng et al. suggested that EA regulates SREBP1 expression, thereby improving insulin resistance, mitochondrial dysfunction, and oxidative stress in PCOS-like animals [13]. These studies provide novel insights into the mechanisms of EA in PCOS; however, further studies are needed to confirm the findings.

EA and MA are both widely used in clinical practice; interestingly, studies on PCOS animal models demonstrate that the mechanism of their action is not identical. Feng et al. demonstrated that EA regulates neuroendocrine and reproductive functions through the endogenous opioid receptor system and manual stimulation by regulating steroid hormone receptors [25]. Johansson et al. reported that MA has a greater effect on glucose tolerance than EA [27]. EA reduces the weight of the subcutaneous fat depot, increases the weight of the soleus muscle, and affects the expression of genes and proteins related to the insulin signaling pathway in the soleus skeletal muscle, while MA improves systemic glucose tolerance and affects gene expression in mesenteric adipose tissue [27]. Benrick et al. further reported that EA has stronger effects on glucose uptake than MA and that it induces more pronounced changes in molecular pathways and improves insulin sensitivity more rapidly, and both EA and MA are equally effective during the poststimulation period [29]. The underlying mechanism of the different actions remains to be elucidated [29].

Different acupoint protocols are employed in studies, and several studies have investigated the different actions. Xu et al. demonstrated that there was no significant difference in body weight when stimulating ST36, SP6, and CV4 separately or in combination. Electrostimulation with ST36 or CV4 alone significantly decreased the T level compared with stimulation with SP6 or their combination. Expression of androgen receptor decreased significantly in the SP6 and CV4 stimulation groups [39]. ST36 significantly improves hormone levels and the expression of receptors in ovarian tissue, but it does not reduce the number of growing follicles. CV4 can regulate follicular development and hormone levels but has no obvious effect on the expression of gonadotropin receptors. The combination group had no evident advantage compared with the single acupoint group [41]. It suggests that the effect of EA at multiple points may not be better than that of a certain empiric point. Whether there is an antagonistic effect on the therapeutic effect of different acupoints is worthy of further study.

### 4.2. Limitations

The positive findings of acupuncture in PCOS animals should be interpreted with great caution since there were several limitations in the present systematic review. First, the substantial heterogeneity should be taken into consideration. Although we performed sensitivity analysis and subgroup analysis, the reason for the generated high heterogeneity was not identified. The difference between acupuncture protocols and different methods used to induce the PCOS model might contribute to the high heterogeneity. Second, the result of the risk of bias assessed by SYRCLE ROB indicated the methodological weakness of the included studies. A majority of the included studies did not report details of sequence generation, baseline characteristics, allocation concealment, randomizing, blinding, or random outcome assessment, which impaired the power of the evidence generated from the present systematic review.

The main implications for further research are as follows: first, the design of the experiment should follow SYRCLE to minimize the risk of bias; second, the report of acupuncture on PCOS animals should follow the Standards for Reporting Interventions in Controlled Trials of Acupuncture (STRICTA) to prompt better quality reporting on acupuncture interventions and help the interpretation and analysis and enable research replications.

## 5. Conclusions

The main strengths of this study are that we systematically reviewed acupuncture experiments in PCOS animal models and performed a meta-analysis, which indicated that acupuncture might have the potential to restore hormone levels. Unfortunately, we could not draw a definite conclusion due to the methodological weakness of the included studies and the high heterogeneity. Well-designed studies are needed in the future to fill this gap.

## Figures and Tables

**Figure 1:** Flow diagram of the study selection process for this systematic review and meta-analysis.

**Table 1:** Characteristics of included studies.

Study ID	Species (Na/Nc)	Randomised	Weight (g)	Model	Acupuncture (acupoints)	Course of treatment	Stimulation parameters	The main outcomes	Result
Stener-Victorin (2003) [18]	SD rats (8/8)	Not reported	195–210	EV	Bilateral in the mm biceps femoris and erector spinae, in somatic segments corresponding to the innervation of the ovaries	Every second or third day, 25 min, 12 times	EA (2 Hz), 1.5 mA	Endothelin-1	*P* < 0.05
Mannerås (2008) [19]	Wistar rats (11/12)	Y	Not reported	DHT	ST29, SP6, in somatic segments that correspond to the innervation of the ovaries	15 min in week 1, 20 min in weeks 2–3, and 25 min, thereafter, 4–5 weeks	EA (2 Hz), 0.8–1.3 mA	BW	NS
Peng (2008) [20]	Wistar rats (11/12)	Y	250 ± 20	TP	ST36, ST40, ST25, SP6	30 min a day, 14 days	EA (2 Hz)	BW FINS	*P* < 0.01 *P* < 0.05
Zhang (2008) [21]	SD rats (14/13)		Not reported	DHT	RN3, RN4, SP6, EX-CA1	15 min, once a day, 6 weeks	MA	T	*P* < 0.01
Zhang (2009)_1 [22]	SD rats (NR)		Not reported	DHT	RN3, RN4, SP6, EX-CA1	15 min, once a day, 6 weeks	MA	T	*P* < 0.01
Zhang (2009)_2 [23]	SD rats (11/12)	Y	Not reported	DHEA	CV4, CV3, SP6, EX-CA1	15 min a day, 5 days	MA	T	*P* < 0.05
Johansson (2010) [23]	Wistar rats (11/12)	Y	299 ± 6; 287 ± 5	DHT	Two needles bilaterally in the abdominal muscles, and two needles were placed in each soleus and gastrocnemius hindlimb muscle, in somatic segments corresponding to ovarian innervations	15 min in week 1, 20 min in weeks 2 and 3, and 25 min thereafter, 5 days/week, 4–5 weeks	EA (2 Hz), 0.8–1.4 mA	WB Glucose infusion rate	NS *P* < 0.001
Feng (2012) [24]	Wistar rats (8/8/8)	Y	Not reported	DHT	Bilaterally in the rectus abdominis and triceps surae muscles at points in somatic segments corresponding to the innervation of the ovaries	15 min in wk 1, 20 min wks 2–3, and 25 min thereafter, 20–25 treatments	EA (2 Hz), 0.8–1.4 mA; MA	T LH	NS NS
Li (2012) [25]	SD rats (9/10)	Y	50 ± 10	DHEA	BL23, RN6, PC6, ST36, SP6, EX-CA1	30 minutes a day, 6 estrous cycles	EA	T LH	Not reported
Johansson (2013) [26]	Wistar rats (10/10/10)	Y	252.8 ± 12.9; 256.4 ± 15.8; 252.3 ± 23.7	DHT	Two needles inserted in the rectus abdominis, and one in triceps surae muscles bilaterally	15 min in week 1, 20 min in weeks 2 and 3, and 25 min thereafter, 5 days/week, 4–5 weeks	EA (2 Hz); MA	BW	*P*=0.29 *P*=0.70
Sun (2013) [27]	SD rats (10/10)	Y	200 ± 20	Letrozole	CV4, CV3	20 min a day, 14 consecutive days	EA (2 Hz), 2 mA	T	*P* < 0.01
Benrick (2014) [28]	Wistar rats (12/12)	Y	Not reported	DHT	ST27, ST28, ST29, SP6, SP9	45 min, single session	EA (2 Hz), 0.8–1.2 mA; MA	Glucose infusion rate	*P* < 0.01 *P* < 0.001
Lai (2014) [29]	SD rats (8/8)	Y	Not reported	TP + high fat diet	RN12, CV4, ST25	30 minutes, 3 times a week, 6 weeks	EA (2 Hz)	HOMA-IR FINS	*P* < 0.05 *P* < 0.05
Chen (2015) [30]	SD rats (10/10)	Y	Y	Prasterone Sulfate + high fat diet	EX-B3, SP6	20 minutes, 5 times a week, 8 weeks	EA (2 Hz), 1.5 mA	T HOMA-IR	*P* < 0.05 *P* < 0.05
Maliqueo (2015) [31]	Wistar rats (10/10)	Y	Not reported	Letrozole	Two needles bilaterally in the abdominal muscles, and two needles were placed in each soleus and gastrocnemius hindlimb muscle, in somatic segments (Th 10- L2) corresponding to ovarian innervations	15 min in week 1, 20 min in weeks 2 and 3, and 25 min thereafter, 5 days/week, 5–6 weeks	EA (2 Hz), 0.6–1.4 mA; MA	T	*P* < 0.05
Zheng (2015) [32]	SD rats (10/10)	Y	45–50	TP + high fat diet	(1) CV12, CV4, SP6; (2) ST36, Hou Hui	20 minutes, 5 times a week, 5 weeks, 2 sets of acupoints alternatively	EA (2 Hz)	T FINS HOMA-IR	*P* < 0.05 *P* < 0.01 *P* < 0.01
Lai (2016) [33]	SD rats (10/10)	Y	Not reported	DHEA + high fat diet	RN4, RN12, ST25	30 minutes, 3 times a week, 5 weeks	EA (2 Hz), 1 mA	HOMA-IR FINS	*P* < 0.05 *P* < 0.05
Li (2016) [34]	SD rats (7/7)	Y	Not reported	DHEA	RN4, SP6, EX-CA1, RN3	15 min in week 1, 20 min in weeks 2 and 3, and 25 min thereafter, 5 days/week, 5 weeks	EA (2 Hz)	HOMA-IR	*P* < 0.05
Lin (2016) [35]	SD rats (6/6)	Y	Not reported	Letrozole + high fat diet	(1) RN4, SP6; (2) BL18, BL20, BL23	15 minutes, 20 days	MA	T HOMA-IR	*P* < 0.01 *P* < 0.05
Maliqueo (2017) [36]	Wistar rats (9/8)	Y	Not reported	Letrozole	Two needles bilaterally in the abdominal muscles, and two needles were placed in each soleus and gastrocnemius hindlimb muscles, in somatic segments (Th 10- L2) corresponding to ovarian innervations	15 min in week 1, 20 min in weeks 2 and 3, and 25 min thereafter, 5 days/week, 5–6 weeks	EA (2 Hz), 0.6–1.4 mA; MA	FINS	NS
Meng (2018) [37]	SD rats (8/8)	Y	Not reported	TP + high fat diet	SP6, RN4, RN12, LI10, ST36	30 min, 5 times a week, 5 weeks	EA (2 Hz)	WB	*P* < 0.01
Xu (2018) [38]	SD rats (10/10)	Y	160 ± 20	Letrozole	ST36, SP6, CV4	20 min, 14 consecutive days	EA (2 Hz), 1–3 mA	WB T	*P* < 0.05 *P* < 0.01
Shi (2019) [39]	SD rats (10/10)	Y	180 ± 20	Letrozole	CV3, CV4	20 min, 14 consecutive days	EA (2 Hz), 2 mA	T	*P* < 0.05
Xu (2019) [40]	SD rats (10/10)	Y	160 ± 20	Letrozole	ST36, SP6, CV4	20 min, 14 consecutive days	EA (2 Hz)	LH LH/FSH	*P* < 0.01 *P* < 0.01
Yu (2019) [41]	SD rats (10/10)	Y	180–200	Letrozole	LI 10, ST36, SP6, RN4	20 minutes, 27 days	EA (2 Hz)	T	*P* < 0.01
Zhou (2019) [42]	SD rats (10/10)	Y	Not reported	Letrozole	CV3, CV4	20 minutes, 14 days	EA (2 Hz), 2 mA	T	*P* < 0.01
Xu (2020) [14]	SD rats (10/10)	Y	160 ± 20	Letrozole	CV3 and the point 5 mm next to CV3 at the same horizontal axis	20 minutes, 14 days	EA (2 Hz), 2 mA	WB T LH AMH	*P* < 0.05 *P* < 0.01 *P* < 0.01 *P* < 0.01
Huang (2020) [43]	SD rats (7/7)	Y	130–170	Letrozole	SP6, LR 3	20 minutes, 14 days	EA (2 Hz), 2 mA	T LH AMH	*P* < 0.05 *P* < 0.05 *P* < 0.05
Kuang (2020) [44]	SD rats (8/8)	Y	50 ± 5	DHEA	RN3, RN4, EX-CA1, SP6	15 min in week 1, 20 min in weeks 2 and 3, and 25 min thereafter, 5 days/week, 5 weeks	EA (2 Hz)	WB	*P* < 0.05
Peng (2020) [13]	SD rats (6/6)	Not reported	Not reported	DHEA	ST29, SP6	15 min in week 1, 20 min in weeks 2 and 3, and 25 min thereafter, 5 days/week, 5 weeks	EA (2 Hz), 0.8–1.3 mA;	T LH LH/FSH	*P* < 0.001 *P* < 0.001 *P* < 0.001
Tong (2020) [45]	Wistar rats (11/14)	Y	Not reported	DHT	ST29, SP6	30 min a day, 5 days a week, 4 weeks	EA (2 Hz), 2 mA	Weight	*P* < 0.001

Na = number in acupuncture group; Nc = number in control group; Ev = estradiol valerate; DHT = dihydrotestosterone; BW = body weight; NS = not significant; FINS = fast insulin; TP = testosterone propionate; DHEA = dehydroepiandrosterone; DHT = Dihydrotestosterone; AMH = anti-Mullerian hormone.

**Table 2:** SYRCLE risk of bias tool for included studies.

Study ID	1	2	3	4	5	6	7	8	9	10	Total
Stener-Victorin (2003) [18]	U	Y	U	Y	U	U	U	Y	Y	Y	5Y5U
Mannerås (2008) [19]	U	Y	U	Y	U	U	U	U	Y	Y	4Y6U
Peng (2008) [20]	U	Y	U	Y	U	U	U	Y	Y	Y	5Y5U
Zhang (2008) [21]	U	U	U	U	U	U	U	Y	Y	Y	3Y7U
Zhang (2009)_1 [22]	U	U	U	U	U	U	U	Y	Y	Y	3Y7U
Zhang (2009)_2 [23]	U	U	U	U	U	U	U	Y	Y	Y	3Y7U
Johansson (2010) [23]	U	Y	U	Y	U	U	U	Y	Y	Y	5Y5U
Feng (2012) [24]	U	U	U	Y	U	U	U	Y	Y	Y	4Y6U
Li (2012) [25]	U	U	U	Y	U	U	U	Y	Y	Y	4Y6U
Johansson (2013) [26]	U	Y	U	Y	U	U	U	Y	Y	Y	5Y5U
Sun (2013) [27]	U	Y	U	Y	U	U	U	Y	Y	Y	5Y5U
Benrick (2014) [28]	U	U	U	U	U	U	U	U	Y	Y	2Y8U
Lai (2014) [29]	Y	Y	U	Y	U	U	U	Y	Y	Y	6Y4U
Chen (2015) [30]	Y	Y	U	Y	U	U	U	Y	Y	Y	6Y4U
Maliqueo (2015) [31]	U	U	U	Y	U	U	U	Y	Y	Y	4Y6U
Zheng (2015) [32]	U	Y	U	Y	U	U	U	Y	Y	Y	5Y5U
Lai (2016) [33]	Y	U	U	Y	U	U	U	Y	Y	Y	5Y5U
Li (2016) [34]	U	U	U	U	U	U	U	Y	Y	Y	3Y7U
Lin (2016) [35]	U	U	U	U	U	U	U	Y	Y	Y	3Y7U
Maliqueo (2017) [36]	U	U	U	Y	U	U	U	Y	Y	Y	4Y6U
Meng (2018) [37]	U	Y	U	Y	U	U	U	Y	Y	Y	5Y5U
Xu (2018) [38]	Y	Y	U	Y	U	U	U	Y	Y	Y	6Y4U
Shi (2019) [39]	U	Y	U	Y	U	U	U	Y	Y	Y	5Y5U
Xu (2019) [40]	Y	Y	U	Y	U	U	U	Y	Y	Y	5Y5U
Yu (2019) [41]	Y	U	U	Y	U	U	U	Y	Y	Y	5Y5U
Zhou (2019) [42]	U	U	U	Y	U	U	U	Y	Y	Y	4Y6U
Xu (2020) [14]	U	Y	U	Y	U	U	U	Y	Y	Y	5Y5U
Huang (2020) [43]	U	U	U	Y	U	U	U	Y	Y	Y	4Y6U
Kuang (2020) [44]	U	U	U	Y	U	U	U	Y	Y	Y	4Y6U
Peng (2020) [13]	U	U	U	Y	U	U	U	Y	Y	Y	4Y6U
Tong (2020) [45]	U	Y	U	Y	U	U	U	Y	Y	Y	5Y5U

Y = yes; N = no; U = unclear. 1: sequence generation; 2: baseline characteristics; 3: allocation concealment; 4: random housing; 5: blinding; 6: random outcome assessment; 7: blinding; 8: attrition bias; 9: reporting bias, and 10: other biases.

**Table 3:** Quality of evidence assessment.

Certainty assessment							No. of patients		Effect		Certainty	Importance
No. of studies	Study design	Risk of bias	Inconsistency	Indirectness	Imprecision	Other considerations	Acupuncture	Control	Relative (95% CI)	Absolute (95% CI)		
HOMA-IR												
6	Randomised trials	Not serious	Serious^a^	Serious^b^	Serious^c,d^	None	51	51	—	SMD 1.28 lower (2.77 lower to 0.22 higher)	⨁◯◯◯ Very low	Critical
T												
8	Randomised trials	Not serious	Serious^a^	Serious^b^	Serious^c^	None	87	84	—	SMD 2.18 lower (3.42 lower to 0.94 lower)	⨁◯◯◯ Very low	Critical
LH												
9	Randomised trials	Not serious	Not serious	Serious^b^	Serious^c^	None	94	91	—	SMD 0.71 lower (1.27 lower to 0.15 lower)	⨁⨁◯◯ Low	Important
LH/FSH												
7	Randomised trials	Not serious	Not serious	Serious^b^	Serious^c,d^	None	68	65	—	SMD 0.59 lower (1.29 lower to 0.12 higher)	⨁⨁◯◯ Low	Important
FBG												
6	Randomised trials	Not serious	Not serious	Serious^b^	Serious^c,d^	None	54	57	—	SMD 0.02 lower (0.8 lower to 0.75 higher)	⨁⨁◯◯ Low	Important
FINS												
7	Randomised trials	Not serious	Serious^a^	Serious^b^	Serious^c,d^	None	62	65	—	SMD 1.46 lower (3.39 lower to 0.48 higher)	⨁◯◯◯ Very low	Important
BW												
4	Randomised trials	Not serious	Serious a	Serious^b^	Serious^c,d^	None	44	48	—	SMD 1.67 lower (4.04 lower to 0.7 higher)	⨁◯◯◯ Very low	Important

GRADE: Grading of Recommendations, Assessment, Development and Evaluation; CI: confidence interval; SMD: standardized mean difference. ^a^I values exceed 75%. ^b^Different animal modelling methods; differences in treatment cycle and dosage; physiological and pathological differences between rodents and humans. ^c^Small sample size. ^d^95% CI included one.

## Data Availability

The datasets supporting the conclusions of this article are included within the paper.
